This article has been retracted.

# Development Mode of Recreation Belt around the City: Ecological Authenticity or Fashion Creativity?

**DOI:** 10.1155/2022/9292668

**Published:** 2022-06-23

**Authors:** Liang Zhao, Yuanyuan Shen, Nailin Gu, Jingyu Dai

**Affiliations:** ^1^School of Humanities, Han-Liang Cultural Research Center, Shangqiu Normal University, Shangqiu 476000, Henan, China; ^2^School of Engineering Management and Real Estate, Henan University of Economics and Law, Zhengzhou 450000, Henan, China; ^3^College of Management, Suqian University, Suqian 223700, Jiangsu, China; ^4^College of Art Design and Media, Sanda University, Shanghai 201209, China

## Abstract

The recreational belt around the city has low population density, good ecological environment, and rich natural and cultural landscapes, which can meet the tourism needs of urban residents to get close to nature and experience culture. Particularly in today's increasingly normal epidemic prevention and control, outing and microtourism have become the first choice of urban public tourism and an important part of rural tourism development. In the process of developing rural tourism, there are two distinct voices: one is to pay attention to the local complex and strive to let people “see mountains and water and remember nostalgia.” In the era of cultural tourism integration, we should promote rural tourism with culture, highlight rural culture with rural tourism, and give full play to the bridge between cultural tourism and rural cultural innovation. In view of this situation, this paper discusses the theme orientation of the advanced development of the recreational belt around the city through three studies. In Study 1, tourists' perceptions of local complex and rural cultural creation were compared through field investigation. In Study 2, brand trust was used as a calibration variable to further test the robustness of the conclusion. Study 3 analyzed the “distortion” mechanism of rural cultural creation and tested the intermediary effect of psychological distance. At the same time, it discusses the evolution model of the recreational space system around the city. The development of recreation space shows that the recreation space around the city is the product of the agglomeration of population and economic activities, and its occurrence and development process is closely related to the expansion of urban space and the change of human living space. This paper analyzes the spatial process of the development of recreation around the city, focuses on the types of recreation space that continue to appear in the development and evolution of modern recreation space, and then tries to find the context of the gradual development and evolution of recreation around the city with the process of urbanization and excavate the organic connection between the recreational space and the city and its surrounding areas in the process of development and evolution. It is found that (1) tourists' perception of local culture is further distorted, which leads to a further reduction in tourists' perception of “local culture” and “recreation,” and (2) the increase in psychological distance is the key psychological mechanism for tourists to perceive “lost property.”

## 1. Introduction

Rural rejuvenation makes use of its market and resource advantages to provide a good environment and major opportunities for tourism-driven urban rural integration for suburban villages [1]. Since 2019, coronavirus disease has had a significant impact on tourism. Under the background of normal prevention and control, the development model of tourism has been reshaped [2]. Under the influence of the radiation effect of the city on the rural revival and the epidemic on the “microvacation” of tourists, the suburbs and surrounding leisure belts around the city have become important tourist destinations. At present, there is an urgent need to improve the quality of travel around residents and improve their happiness in tourism [3]. The basic theory of fractional calculus and its application based on practical schemes and methods are provided and illustrated with applicable engineering and technical examples, with particular emphasis on the design of fractional-order controllers [4].

Microvacations are usually centered around metropolitan areas where travelers live and seek destinations within a two-hour drive. Tourists give up long-distance travel because they need to prepare various things for long-distance travel. In order to avoid time-consuming preparation, they choose short-distance travel. As the main way of travel, cities and towns use their leisure time on weekends to stay away from the mundane noise, integrate into Acadia, and seek a balance between work and life. Energy consumption and time consumption are lightweight, but this does not mean that the cost is low. People pursue new experiences, cultural acquisition, happiness of family participation, refinement of basic needs such as catering and accommodation, so that tourists can deeply experience the culture and life around them. In the process of microvacation in the suburbs of the city, the tourists pursue the ecological original local complex, or the rural cultural creation with fashionable taste, which is not only related to the tourist satisfaction but also related to the healthy and sustainable development of rural tourism. In view of this, this paper explores the impact of different development models on the industry and the psychological mechanism behind them through four researches and uses brand trust as an indicator variable to provide a more complete chain of evidence. Finally, the differences in model “distortion” in different image enterprises are clarified.

## 2. Theoretical Basis and Literature Review

### 2.1. Ring-City Recreation Belt and Urban Microtourism

Re BAM around the city originally refers to the leisure gathering space around the metropolis. Since the 1990s, it has become a normal life for urban residents to use their holidays for short-distance tourism and recreational activities. Urban leisure activities form a cluster in cities of different levels and population sizes [5].

Urban residents are the most important source of tourists. Particularly on holidays, leisure activities in the surrounding areas of the city have maintained a rapid growth momentum for a long time, which confirms the driving role of big cities [6]. Most of the existing studies on the recreational belt around the city take supply and spatial structure as the starting point and generally pay attention to the concept and causes, spatial structure and temporal and spatial evolution, recreational land types, and resource evaluation of the recreational belt around the city. The case studies gradually expand from large cities to small- and medium-sized cities with different population sizes. With the implementation of the rural revitalization strategy and the surge of outings and surrounding tourism under the background of epidemic prevention and control, the demand of urban residents for near urban recreation has attracted people's attention, but it is not enough to explore the recreational belt around the city from the perspective of demand [7]. According to the analogy and metaphor of the energy band models of organic and inorganic semiconductors, the coupling relationship is established. The transconductance before and after bending predicted by the derived analytical model is in good agreement with the data measured by DNTT-based OFET-bending experiments [8]. Traditional market research focuses on the investigation and analysis of residents' recreational behavior characteristics and preferences, rarely involves the exploration of the causal relationship between urban residents' psychological consciousness and recreational behavior in near urban areas, and fails to reveal the decision-making mechanism and process of leisure behavior.

### 2.2. Local Complex and Rural Cultural Creation

Nostalgia is people's unforgettable memory and lingering attachment to their hometown. Rural tourism is essentially traveling in the “rural concept.” Rural space actually provides tourists with the semantic field of rural imagination. Rural areas are the hometown where people touch tradition and cultivate their hearts. Pastoral songs express people's sincere admiration for the original state, the ardent longing for the free state, the self-construction of the distant state, and the natural transformation of the cosmic state. Tourists travel in the countryside, using symbolic rituals or processes to comfort the repressed and alienated mind. Therefore, the nostalgic experience of traditional village tourists should be improved from the aspects of nostalgic cultural landscape protection, nostalgic tourism market segmentation, and experience tourism product development [9]. An optimization problem is solved by a genetic algorithm (GA) to minimize the cost function in a small region around the initial parameters of FOPID (optimal design of discrete-time fractional-order PID controller for idle speed control of an IC engine 2020). Compared with the experimental data, it is found that, compared with the traditional DD model, the Fr-DD model can obtain more accurate transconductance prediction, especially in the subthreshold and low gate source voltage regions of OFET [10].

The competitor's view is that “country” plays an important role in urban and rural tourism and cultural integration and should promote the development of regional characteristic economy and tourism through the development of country and industry [11]. “Rural cultural innovation,” as an important way for cultural creativity to realize rural revitalization, is the innovative application of strategic thinking and implementation path of cultural creativity in rural revitalization. The logical starting point of “rural cultural innovation” is rural cultural resources. Through the evaluation of rural cultural value and the transformation of rural cultural capital, we can create cultural products and services with rural characteristics and then realize the optimal exchange of rural value through the rural cultural market. With the support of rural cultural policies, it will eventually develop into rural characteristic cultural industry and rural characteristic cultural economy. The breakthrough of rural cultural construction lies in innovation. Innovation should be guided by adjusting measures to local conditions, coordinate economic and cultural development and urban and rural cultural development, adhere to the combination of inheritance and innovation, and give consideration to the leading role of the government and the dominant position of farmers.

## 3. Research Design

### 3.1. Periurban Rural Tourism and Tourists' Perceived Value

The accurate positioning and reasonable planning of recreation belts all over the country can improve the quality of public recreation and help to promote the adjustment of rural industrial structure. The recreational belt has become the most suitable leisure destination for residents all over the country, and recreational activities have also become a way of urban leisure [12]. Leisure agriculture and rural tourism are the “trinity” of agricultural tourism culture, the synchronous improvement of production and living ecology, and the deep integration of rural primary, secondary, and tertiary industries. The fidelity of 2D MSD structure in inverted interleaved TFT modeling is verified, and a new modeling method is developed, which can be extended to other types of flexible thin-film transistors [13]. “Local complex” reflects the spiritual and cultural characteristics of the Chinese people, is also the unconscious inheritance of the collective memory of the Chinese people, and deeply interprets the tension of “cultural intimacy” between tourists and society. Based on this, the following assumptions are put forward:

  H1: compared with local complex, rural cultural creation has a lower perceived value for tourists.

### 3.2. Mediating Effect of Psychological Distance

Psychological distance refers to the distance between the stimulus and self perceived by people at this time. From a philosophical point of view, Bloch's theory establishes a binary interaction between subject and object but fails to solve the problem of their coexistence [14]. Under the special background of the rebound of the epidemic, most people are forced to “limit traffic,” “limit flow,” or “stay at home” for a long time, which objectively leads to psychological changes of some people. They actively and timely carry out psychological screening and evaluation for different groups in the early stage and take TCM psychological prevention and treatment technology for intervention so as to reduce the psychological harm and secondary harm caused by the epidemic [15]. With the local rebound of the epidemic, the psychological state of anxiety, anxiety, tension, panic, and vigilance will continue to exist. With the gradual recovery of domestic tourism in the postepidemic era, it is particularly important to help tourists adjust their negative psychology, enhance their sense of security, and shorten the psychological distance between tourists and destinations through effective ways. This paper selects the social distance in the psychological distance as the measurement dimension to pay attention to the closeness and warmth of urban residents to rural areas in the postepidemic era. Referring to the research of Tang et al., psychological distance is introduced into the research model as an important intermediary variable [16], and the following assumptions are put forward:

  H2: psychological distance plays a mediating role in the impact of rural tourism form on tourists' perceived value.

Based on the above factors, the research model is shown in Figure 1.

### 3.3. Research Framework

Three researches were designed in this paper. In research 1, field investigation was used to compare the differences in the perceived value of rural tourists under the local and cultural and creative modes, and the service “distortion” caused by cultural and creative modes was revealed. In research 2, a scenario experiment was used to further test the robustness of the conclusion of research 1 in a more strictly controlled scenario experiment, and brand trust was added as an indicator variable of tourists' perceived value to provide a more complete chain of evidence. Research 3 analyzed the internal mechanism of “distortion” caused by the cultural creation mode and tested the mediating effect of the psychological distance. The research framework is shown in Table 1.

## 4. Research 1

### 4.1. Experimental Design and Process

In research 1, a single-factor intergroup design (development model: rural versus cultural innovation) was used to compare the differences in perceived service value of rural tourists to local culture and cultural creativity. For the consideration of controllability and convenience, this research was carried out in rural tourist attractions. Compared with laboratory experiments, individual feelings and reactions in field investigation will be closer to reality and have higher reliability. Therefore, research 1 selected an ecological original scenic spot and a cultural creative scenic spot with a similar distance from the main city and ticket price to carry out field investigation. In this research, screening questions were added to the questionnaire to ensure that the survey met the research objectives as much as possible. In the end, a total of 95 tourists from the two scenic spots participated in the survey and filled in the questionnaire upon departure. A total of 85 valid samples were obtained (male 50.7%; *M* age = 38.12; SD = 9.602).

### 4.2. Experimental Results

As for the dependent variable of tourists' perceived service value (*α* = 0.95), the results of one-way ANOVA showed that the perceived value of tourists in the cultural and creative group was significantly lower than that in the ecological and original group (*M* cultural and creative = 5.63, *M* local = 6.19, *F* (1, 78) = 5.399, and *P*=0.019). Covariance analysis was further used to test the influence of different modes on perceived service value when the age and gender of the subjects were controlled, and the results were consistent with one-way ANOVA. Age has no significant influence on tourists' perceived value (*F* (1, 76) = 2.499; *P*=0.129), and gender has no significant influence on tourists' perceived service value (*F* (1, 76) = 0.096; *P*=0.761). Subsequent researches have controlled the gender and age of the samples, and the analysis results show that the influence is not significant. H1 was supported in research 1.

### 4.3. Discussion

In research 1, field investigation was used to preliminarily prove that, compared with traditional ecological authenticity, cultural and creative tourists' perceived value was lower; that is, service “distortion” existed. The potential risk of research 1 is that, in addition to the differences in local culture and cultural creativity, there may also be differences in brands, geographical locations, and other factors between the two scenic spots selected for on-site investigation. In addition, the environmental atmosphere of scenic spots, such as catering, accommodation, entertainment, and other factors, may also affect the level of tourists' perceived value. Therefore, under the mode of improving cultural creativity, the survey results of tourists' perceived service value are still at a high level. Therefore, the scenario simulation experiment of the same scenic spot will be adopted in research 2 to test the research hypothesis again after controlling factors such as brand and geographical location as much as possible.

## 5. Research 2

### 5.1. Experimental Design and Process

In research 2, a single-factor intergroup design (service model: ecological authenticity versus cultural creativity) was used to test the distortion effect of cultural creativity through situational experiments. At the same time, a large number of previous researches have proved that tourists' perceived value can affect tourists' brand trust therefore, brand trust was selected as the criterion variable in this research for joint testing to enhance the robustness of test results.

In the experiment, “A” agricultural carnival official promotional video was selected as the original video material, and the footage of ecological authenticity and cultural creativity was, respectively, cut into two 30-second video materials. The two videos contain relatively complete service processes. Since they are the same rural tourism scenic spots, the overall style, music background, and video protagonists are consistent so that the potential interference factors can be controlled as much as possible. The experiment recruited 90 students (male 35.3%; *M* age = 20.21; SD = 3.399). Participants were randomly divided into two groups. The “cultural and creative group” was told to watch a rural tourism cultural and creative video, while the “ecological and true group” was only told to watch a rural tourism video. They were asked to fill in a questionnaire after watching the video material.

### 5.2. Experimental Results

The results of one-way ANOVA showed that there was a significant difference between groups in perceived value level of tourists (*α* = 0.82) (*M* cultural innovation = 5.48, *M* local = 6.10, *F* (1, 85) = 10.298, and *P*=0.003), and H 1 was verified. For brand trust (*α* = 0.83), the difference between groups was also significant (*M* cultural innovation = 5.49, *M* local = 6.01, *F* (L, 85) = 11.301, and *P*=0.002). In the independent variables, the mode of “ecological authenticity” was further set as “0,” and the mode of “fashion creativity” was set as “1” (the same as in researches 3 and 4). Bootstrap method was adopted to test the mediating effect of tourists' perception of service warmth (PROCESS, Model 4, sample size 5000, confidence interval 95%). The results showed that the mediating effect of tourists' perception of service warmth was significant (*β* = −0.45, LLCI = −0.782, and ULCI = −0.179, excluding 0). After controlling the mediating variables, the service model has no significant effect on brand trust (LLCI = −0.261 and ULCI = 0.081, including 0), proving that psychological distance plays a complete mediating role.

### 5.3. Discussion

For the same scenic spots in the rest zone around the city, compared with the ecological authenticity, tourists not only have a lower level of perceived value in the face of fashion creativity but also have lower trust in the brand. Research 2 retested the influence of fashion creative mode on tourists' perceived value in the ring-city rest zone in a scenario experiment with stricter control and extended the evidence chain through brand trust, which provided stronger evidence for the research conclusion. In research 2, participants' perceived value was generally at a high level in both the ecological and creative scenes due to the influence of the overall tone of the promotional film and the emotion of the protagonist in the promotional film. In addition, research 2 takes university students as research objects, which cannot completely represent the perceived value level of tourists. In order to eliminate the influence of the above factors, research 3 used social samples and text materials to conduct intragroup experimental manipulation. Under more strict control conditions, we examine the “distortion” effect of cultural creativity, examine the mediating effect of psychological distance, and deconstruct the psychological mechanism of the “distortion” phenomenon.

## 6. Research 3

### 6.1. Experimental Design and Process

In research 3, an intragroup experimental design was adopted (scenic spot model: ecological authenticity versus cultural creativity), and “W” Town, which advocates returning to rural areas and experiencing slow rural life, was selected as experimental material. Each participant took part in two experiments, 24 hours apart. In order to control the influence of video tone and hero's emotion on participants' perception of service value, this research used text material to describe the situation. Participants were asked to fill in the same questionnaire after each reading and leave the last 4 digits of their mobile phone number for data matching. It is the first time to present the brand image of W Town and relevant text materials of the service process for participants. For the second time, participants were informed in the experimental materials that, in order to conform to the development of The Times and industry, W Town began to implement the fashion cultural and creative mode. If the comparison of the two measurement results shows that the level of perceived service value of tourists in the second experiment significantly decreases, then the “distortion” effect of the fashion cultural creation mode is verified. Therefore, an in-group experiment was designed to control the relationship between participants and brands. The experiment recruited 50 participants (56.3% male; *M* age = 36.12; SD = 6.409).

The text materials used in the experiment are as follows:

  The first text (from the introduction, excerpted text):
  The town is built on the basis of water. It skillfully uses idle land and the past free pit. With its unique natural environment and rich ecological resources, it integrates characteristic agriculture, rural tourism, and local folk customs. Throughout the year, you can experience unique folk culture scenes so that you can improve the fun of life in the environment of traditional culture.
  The second written materials:
  In order to conform to the trend of the times, W town began to pursue fashion culture and creative business model. Through multidimensional perspectives, it explored and refined the rural culture and spiritual culture at the core of “local” and constructed and interpreted the theme of rural cultural image and characteristic brand, so as to form a unique personalized, storytelling, and IP derivative system of rural tourism.

### 6.2. Experimental Results

*T*-test results of paired samples showed significant differences in the perceived warmth level of tourists (*α* = 0.93) (*M* for the first time = 5.89, *M* for the second time = 3.99, *T* (49) = 5.79, and *P* < 0.001), and H1 was verified again. Similarly, for psychological distance, paired sample *T*-test results also showed significant differences (*M* first = 4.69, *M* second = 2.78, *T* (49) = 7.01, and *P* < 0.001). Bootstrap method was used to test the mediating effect of psychological distance (PROCESS, Model 4, sample size 5000, confidence interval 95%). The results showed that psychological distance had a significant mediating effect (*β* = −0.779, LLCI = −1.320, and ULCI = −0.381, excluding 0). After controlling the mediating variables, service mode still had a significant impact on tourists' perception of service warmth (*β* = −1.110, LLCI = −1.799, and ULCI = −0.389, excluding 0), proving that psychological distance played a partial mediating role and H2 was verified.

### 6.3. Discussion

Research 3 verifies the mediating role of psychological distance in the influence of fashion creative mode on “distortion” through text manipulation and analyzes the “distortion” mechanism of rural tourism fashion creativity. Li and Zhao [17] showed that, under the background of the epidemic, the psychological carrying capacity of outdoor scenic spots based on tourists has changed. The study found that wearing masks has significant interactive and main effects on congestion norms. Wearing masks can shorten the psychological carrying capacity of tourists. discussed the rural tourism intention in the epidemic era. The results show that the relationship between tourists and destinations, trust, and common vision can shorten the psychological distance between tourists and destinations. The epidemic not only caused great losses to the national economy but also brought psychological impacts to tourists. Therefore, the model is analyzed and verified according to the large sample survey data in China during the epidemic period. The results show that tourists' anxiety has a great impact on the recovery of tourism, and the recovery of tourism will significantly and positively affect the willingness to travel.

## 7. Conclusions and Suggestions

### 7.1. Research Conclusions and Theoretical Contributions

In the postepidemic era, considering the cost and safety, rural tourism around the city can recover rapidly with the advantages of low density, close to nature, and short distance. After combining the relevant research literature and predicting the actual situation, combined with the crisis life cycle theory, taking the 2003 SARS epidemic as a comparative case, the evolution process of the tourism epidemic crisis is analyzed. The study found that the epidemic crisis evolution process of the tourism industry can be divided into three stages: short-term sharp reduction stage, medium-term transition stage, and long-term optimization stage, which correspond to the stage characteristics of harm extremes, rebound uncertainty, and the coexistence of opportunities and challenges. On this basis, the short-term rescue strategy, medium-term regulation strategy, and long-term optimization strategy are put forward [18]. Rural tourism has become the first choice for urban residents to relax and enhance parent-child relations. Parent-child tourism has become a dark horse in the tourism market in recent years because it conforms to the characteristics of the higher spiritual pursuit of cultural tourism [19]. In the context of brigade integration, rural tourism promotion should pay more attention to cultivating new business forms of cultural tourism. The coordinated development of rural tourism and cultural industry should pay attention to the symbolization and stage of culture, the branding and visualization of rural areas, and the refinement and diversification of product business forms and realize the benefits of villagers in tourism development and the sustainable development of rural tourism industry [20]. However, it only carries nostalgia and traditional culture, excavates the cultural connotation of local characteristics, avoids the homogenization of rural tourism products, improves the core attraction of rural tourism, and promotes the development of rural tourism quality [21]. This paper reveals the potential risks of cultural creation in rural tourism through three experiments and discusses the decline of perceived service value and its impact on enterprise brand trust when there is a lack of “local” elements in the process of rural tourism. The results show that (1) compared with ecological authenticity, fashion creativity can significantly reduce the perceived service value of rural tourists, that is, service “distortion,” which leads to the decline of tourists' trust in the brand of scenic spots; (2) the increase of psychological distance is the key psychological mechanism for tourists to perceive the decline of service value.

To sum up, the theoretical contributions of this paper are mainly reflected in the following two aspects.

First of all, this paper focuses on the impact of fashion creative mode on the characteristics of rural tourism “ecological authenticity,” a more comprehensive analysis of the impact of cultural creativity on the ring-city recreation belt scenic spots. For recent outings, tourists' perceived value is an important dimension of industry evaluation. Most existing researches focus on the positive role of technology in improving service efficiency and reducing costs from the perspective of capacity and seek ways to promote technology promotion and tourists' acceptance based on this. This paper focuses on the dimension of ecological authenticity, which can better highlight the characteristics of rural tourism, expands the previous single-dimension research from the perspective of ability, and deepens the research topics applied in the field of rural tourism.

Secondly, this paper finds that fashion creativity will bring “distortion” to rural tourism, revealing the “double-edged sword” function of technology. Previous researches generally believe that fashion creativity can bring many advantages such as popularity promotion and efficiency improvement, but this research finds that it will also lead to service “distortion” and threat to brand trust. The conclusion of this research supplements the research on the negative impact of technology and more completely analyzes the impact of technological change on rural tourism. Bringing rural tourism into the development of the recreational belt around the city, taking the rural tourist destination as the point and the recreational belt around the city as the axis, and adopting the development mode of point axis development will drive the whole recreational industry to achieve breakthrough development.

### 7.2. Practical Suggestions

Based on the above research conclusions, we provide the following suggestions for the RBZ scenic spots to help them avoid the “distortion” problem and its negative effects in the process of developing fashion creativity.

First of all, scenic spots in rural areas around cities should not blindly believe in cultural creation. In the process of pursuing the fashion effect brought by cultural creation, they should also pay attention to the possible negative impact of nostalgia. Nostalgia is mainly divided into four dimensions: local perception, functional perception, emotional perception, and real perception. Tourists' local perception, real perception, and functional perception will have a significant impact on emotional perception. In all dimensions of tourists' homesickness, in addition to functional perception, local perception, real perception, and emotional perception will have a significant impact on tourists' loyalty. In the characteristics of tourists' tourism activities, the stay time and tourism experience will affect tourists' homesickness. Residents' nostalgic local perception and functional perception have a significant impact on the dimension of tourists' emotional perception. In all dimensions of homesickness, emotional perception has a negative significant impact on residents' support, functional perception has a significant effect on residents' support, and neither local perception nor real perception has a significant effect on residents' support. Among the residents' living characteristics, living time, participation form, and the number of people participating in tourism will affect residents' support. Tourists and residents have significant differences in emotional perception and true perception in all dimensions of homesickness, but there is no significant difference in local perception and functional perception. In the process of using fashion creativity, we should change the concept and management mode of the scenic spot and find and solve problems according to the specific situation of tourism in the recreational belt around the city. In the development of tourism in the new era, the development of scenic spots should implement the concept of sharing, including not only the sharing of economic interests but also the sharing of spirit. Therefore, this study studies the nostalgia of tourists and residents and its impact effects and puts forward the following suggestions for the realization of host-guest sharing in the scenic spot: protect the style of the ancient town, excavate the local traditional culture, maintain the local authenticity, and improve the tourism service facilities to meet the nostalgia of tourists and increase the loyalty of tourists; improve local infrastructure, enhance residents' participation, and improve living standards to meet residents' homesickness and increase residents' support.

Secondly, local and homesickness factors should be added to solve the “distortion” problem when fashion creativity is applied to the development of tourism in the ring-city recreation belt. Although the fashion creative mode squeezes the element of “ecological authenticity” out of the market, it can highlight the elements of hometown and nostalgia through ingenious transformation and innovative expression. Fashion creativity should be retained in the ring-city recreation belt, and the developers of scenic spots should retain the ecological authenticity to improve customers' perception of homesickness so as to shorten the psychological distance, promote the development of ring-city tourism “ecological authenticity” and “fashion creativity” in parallel, and realize the balanced development of ring-city tourism in two dimensions.

Finally, the scenic spots should pay special attention to solve the “distortion” problem. For such enterprises, the negative impact of cultural creative mode on their local image may greatly destroy their core competitiveness in the market. Therefore, creativity, as the image of the ecological theme of the scenic spot, on the one hand, we should carefully choose whether to adopt the fashion creative mode. On the other hand, if we choose the imported fashion creative mode, we need to consider other schemes at the same time, so as to meet the expectations and needs of tourists for the local area, maintain the local brand image, and ensure that its core characteristics are not weakened.

## 8. Research Limitations and Prospects

The recreational belt around the city has many forms, such as scenic spots, restaurants, hotels, and tourism service centers. This paper has verified this scenario in scenic spots. Secondly, for the impact of “distortion,” this paper only considers brand trust, and whether there are other important tourist psychologies and behaviors affected, such as emotional connection, tourist loyalty, and word of mouth evaluation, and how to solve the possible negative impact of “distortion” need further research and exploration in the future. Thirdly, the main goal of this paper is to prove the “distortion” impact of fashion service mode and the effect of the combination of the decline in the perceived value of service and the increase in perceived service ability on consumers' behavioral intention, which needs to be further discussed in the follow-up research. In addition, it remains to be discussed whether and to what extent the fashion creative mode can improve the ability perception of tourists on the ring-city recreation belt to the local enterprises and whether the local enterprises can improve and renew their image through this mode.

## Figures and Tables

**Figure 1:** Theoretical model.

**Table 1:** Research framework.

Research	Design	Hypothesis	The research situation
Research 1	Development mode: ecology versus cultural	H1	Rural eco-tour and rural cultural and creative tour (site survey and intergroup design)
Research 2	Development mode: ecology versus cultural	H2	The same mode of rural tour (scene experiment and group design)
Research 3	Development mode: ecology versus cultural	H3	Rural ecotourism (scenario experiment and intragroup design)

## Data Availability

The data underlying the results presented in the study are included within the paper.
